This article has been retracted.

# The Influence of Public Mental Health Based on Artificial Intelligence Technology on the Teaching Effect of Business Administration Major

**DOI:** 10.1155/2022/5353889

**Published:** 2022-09-09

**Authors:** Yixia Lu

**Affiliations:** College of Management Science, Chengdu University of Technology, Chengdu 610059, China

## Abstract

As an emerging technology, public mental health based on artificial intelligence engineering has broad application and development prospects in improving teaching effects, realizing high efficiency and intelligence, and improving refined education. The application of public mental health based on artificial intelligence engineering in the practice of the teaching effect of business administration has a very positive significance for accurately discovering the mental health and teaching effect of business administration students. For the sake of improving the teaching effect of business administration major, we come up with a method for the influence of public mental health on the teaching effect of business administration profession based on artificial intelligence engineering. Firstly, we collect the video and audio of the teaching of business administration, conducts data screening and cleaning, and sorts out the video and audio synchronization clips as training data. Secondly, we propose a multimodal feature extraction network and a multimodal fusion network for the extraction and fusion of video and audio clips, respectively. Then, the fully connected network structure is used to evaluate and classify the effect of business administration professional teaching, and use mental health factors for evaluation to avoid human intervention and improve the prediction effect. Finally, through intensive experimental results, we prove that the method raised by us can use artificial intelligence engineering to evaluate the teaching effect of business administration majors from the perspective of public mental health and achieve good experimental results.

## 1. Introduction

The continuous evolution of artificial intelligence has promoted the integration of artificial intelligence engineering and industry, spawned a large number of artificial intelligence models, and changed people's production and lifestyle [1, 2]. Society has rapidly gotten into the era of intelligence, and in many fields, including education, have undergone tremendous changes, and the content, form, and evaluation are constantly changing [3, 4]. Under the backdrop of artificial intelligence engineering, the training of business administration professionals has undergone certain changes, which makes the traditional business administration teaching more incompatible in the era. Exploring new business administration teaching modes, solving traditional business administration major teaching problems, and promoting the teaching reform of business administration have become the top priority [5, 6].

Facing an increasingly turbulent business environment and increasingly fierce competition, many companies use artificial intelligence, deep learning, cloud computing, etc. to optimize their organizational structure, improve operational efficiency, promote management efficiency, and decrease operating costs [7]. Through the internal boundaries and barriers of the organization of data, the circulation and collaboration of the supply chain are optimized, and the individual kinetic energy of the company and employees is stimulated [8, 9]. All the above-mentioned changes and developments are constantly improving and developing the theory and practice of traditional business administration [10, 11]. However, due to various reasons, the current curriculum and teaching of business administration have not kept up with the theory and practice of business management under the wave of digitalization, and the impact on the current subject teaching and student training cannot be concretely reflected. Artificial intelligence technology not only has a profound impact on the teaching of business administration but also promotes the development of teaching to some extent. The technologies represented by artificial intelligence technology and personalized or customized education are constantly expanding teaching methods, enriching teaching forms, and actively exploring the reform ideas and practical ways of applying artificial intelligence engineering to the course content and teaching methods of business administration majors [12, 13].

Although the current artificial intelligence technology has a comprehensive range of applications in the teaching of business administration, these technologies rely on manually selected influencing factors to evaluate the effect of business administration and are easily affected by human factors [14, 15]. In last years, applying artificial intelligence engineering to the field of mental health and evaluating the teaching effect of business administration majors from the field of mental health has become a new solution [16, 17]. Artificial intelligence engineering is a science that investigates and grows methods, technologies, and technique systems for imitating and visualizing human intelligence [18, 19]. Machine learning is the most important technical means of artificial intelligence, which aims to explore and model complex high-dimensional interactions between a large number of variables [20, 21]. Through the acquisition and analysis of data by artificial intelligence engineering, and the use of artificial intelligence methods to express the relationship between modeling features and mental health, intelligent mental health assessment replaces manual assessment to a certain extent, avoiding the elements of human manipulation [22, 23]. The traditional teaching method has been following the fixed talent training mode, teaching students the relevant professional basic knowledge through classes, but the teaching method is too outdated and difficult to adapt to the current era of intelligence. The current teaching methods mainly advocate individualized learning methods, teach students in accordance with their aptitude, and improve students' sense of participation.

To evaluate the teaching results of the business administration major more fairly and justly, we propose an evaluation method for the teaching effect of the business administration major on public mental health based on artificial intelligence technology [24, 25]. We adopt artificial intelligence-based mental health evaluation form and data analysis method, which enables researchers to approach the task scenario in a more simulated way, obtain multimodal data for analysis and modeling, and achieve more efficient and accurate predictions [26, 27]. The application of mental health assessment based on artificial intelligence engineering to the teaching effect of business administration has a comprehensive range of applications, and it has certain conducting significance for the investigation on the teaching effect of business administration and avoids the interference of human factors [28]. The traditional method of evaluating the teaching effect of business administration majors mainly relies on some artificially selected factors for evaluation, which will cause human influence factors, that is to say, to a large extent; it mainly depends on human factors to determine the evaluation effect. Such an evaluation method is unfair and unjust. Therefore, in this paper, the public mental health perspective is adopted to evaluate the effect of learning and avoid human interference.

## 2. Related Work

### 2.1. Public Mental Health

The evolution and expansion of society have accelerated the pace of people's life and intensified the competition in society. These rapid changes have resulted in a huge impact on individual mental health. In the context of this stressful era, how to conduct an efficient and accurate evaluation of mental health is particularly important. How to understand people's mental health status and intervene in advance is the main task. The rapid evolution and utilization of artificial intelligence engineering has spawned the field of public mental health based on artificial intelligence technology. Intelligent mental health can solve the imperfection of traditional methods and reduce the efficiency of missed diagnosis and misdiagnosis, which is of extremely magnitude for the detection of mental health.

Artificial intelligence technology has important applications in the mental health of undergraduates. Firstly, according to the analysis of artificial intelligence technology, teachers can grasp the mental health of the student group. For students with serious mental health problems, they will be the focus of public mental health education in the future. Through the design and implementation of various types of educational guidance or mental health activities, it guides college students to overcome psychological barriers. Mental health assessment, based on the background data recorded in college students, sorts out the common mental health problems such as anxiety and depression among college students and designs related public mental health education activities. So that students can gradually perceive problems and recognize the emergence of problems in continuous learning. Firstly, identify the cause of the problem and gradually overcome mental health problems. Secondly, after the public mental health system based on artificial intelligence obtains students' mental health-related data, it pushes mental health-related test reports for each student and pushes mental health guidance for each student, so that students can know what method they want to use in order to get out of the psychological predicament and achieve good development.

This year, artificial intelligence engineering has been widely used in the business field and gradually deepened into colleges and universities, making many teachers perceive and recognize the practical value of these new technologies. However, few colleges and universities realize that the practice from the perspective of combining technology with the mental health of college students does not pay much attention to this new technology. Firstly, it restricts the application of advanced scientific research results such as artificial intelligence engineering to the practice of public mental health education, which makes the education and teaching model too outdated. Secondly, insufficient attention is paid to artificial intelligence technology, which leads to the lack of relevant support for the application research and practical exploration of artificial intelligence engineering in college students' mental health, and the development of mental health education cannot be promoted.

Artificial intelligence engineering is a universal technology. Numerous research experiments have shown that these preface technologies can be applied to the field of public mental health, especially the mental health of college students. However, there is currently a lack of clear application ideas and mature content guidance, which makes artificial intelligence technology facing greater difficulties in the mental health education of college students. Simultaneously, artificial intelligence engineering in the field of college students' mental health involves artificial intelligence, big data and psychology, and other related majors, which demands researchers not only to have professional knowledge in psychology but also to have artificial intelligence technology, big data technology, and software platform development capabilities. However, professionals in this field are relatively scarce in colleges and universities, which makes the application of artificial intelligence engineering in the field of public mental health very difficult. In addition, although artificial intelligence engineering can improve the pertinence and accuracy of college students' mental health education, this effect needs to provide enough data information to make the model run with accurate data. The participation of undergraduates in public mental health education activities is the premise and foundation of the advantages of artificial intelligence technology. However, at present, the number of college students who actually participate in the activities is relatively small, which makes it impossible to obtain accurate data. The problem of poor participation results in the ineffectiveness of the artificial intelligence technology in the field of college students' mental health, which affects the application of artificial intelligence engineering.

The continuous development of the current society has led to people's life pressure and reduced psychological endurance, which can easily lead to mental health diseases. However, the traditional public mental health assessment methods are inefficient, difficult to detect mental health problems, and easy to cause misdiagnosis. The method based on artificial intelligence technology has high operation efficiency and more accurate assessment of people's mental health.

### 2.2. Teaching Business Administration

The continuous development of artificial intelligence engineering has led to an endless stream of intelligent technologies, which not only changed people's production and lifestyle but also brought a certain affection and impact on the education system. Artificial intelligence technology has provided new ideas for the teaching reform of business administration majors. However, the traditional education and teaching mode is the mainstream pattern of business administration majors teaching remains unchanged. Therefore, in the context of artificial intelligence, the teaching of business administration has ushered in new development opportunities and challenges. In the context of artificial intelligence technology, reforming the teaching of business administration is the trend of the development of ICBC management teaching and education. Relevant researchers actively design strategies to build a new model of business administration teaching to promote the development of business administration teaching. Export more high-efficiency business management competent people for the society.

Problems existing in the instruction mode of business administration profession:

1. The first is that the professional goals of business administration are difficult to achieve. In the context of artificial intelligence, the requirements for high-quality business management talents are getting higher and higher, but there is a lack of relevant testing methods and technologies for students' teamwork ability and mental health evaluation. These problems have led to increasingly prominent contradictions between teachers and students, and it is far from enough to improve students' teamwork ability and mental health assessment through projects as a carrier. Cultivating students' innovative ability means that students need to master more basic knowledge, constantly have their own innovation and tear up, and be able to connect across borders. The cultivation of students' executive ability means that students need to be cultivated through decision-making and execution tests
2. The degree of capacity building needs to be strengthened. A survey was carried out on the talent training of related business administration majors in my country. The results of these related surveys show that the talent training methods in my country's middle and high schools are relatively common. This problem causes students' foreign language skills, computer technology, business management, and other aspects to lag behind the era of artificial intelligence. In the major of business administration, the school's designated ability training plan is mainly realized through course performance. The lack of professional teachers leads to unreasonable guidance for students, which makes it difficult for students to achieve their predetermined goals after the end of education. These problems make it difficult for them to understand specific knowledge, and they have a shallow understanding of business administration in the context of the era of artificial intelligence, and they cannot apply what they have learned
3. The module setting is unreasonable. Colleges and universities have unreasonable module settings for business administration schools and lack more detailed distinctions and definitions for business administration teaching. And the difference between the courses is big, the plates are separated from each other, and there is no clear distinction or definition. There are many modules in the teaching process of business administration, but from the perspective of career development of students, it does not meet their needs for relevant professional knowledge. In the required courses and elective courses, the basic courses of majors are not closely integrated with mental health and core courses, which lead to the incomplete construction of the knowledge system and reduce the actual effect of the whole study. Judging from the current situation, the current stage of business administration majors has a wide variety of teaching modes and a large number of courses, but these courses are independent of each other, which cannot effectively build a complete learning framework, which reduces the overall effect of college students' learning. The improvement needs more attention from colleges and universities

Artificial intelligence technology is a research direction based on deep neural networks. It mainly relies on network models to predict or classify some data indicators and then use these technologies to evaluate the prediction effect of network models. At present, many enterprises use this technology to optimize the structure of the enterprise and improve the performance of the enterprise, so it is feasible to apply this method to the teaching of business administration.

## 3. Methods

The impact model of public mental health based on artificial intelligence technology on the teaching effect of business administration majors proposed in this paper is mainly composed of five parts: video and audio collection, audio feature extraction, video feature extraction, multimodal fusion, and business administration major. Teaching effectiveness evaluation: The video and audio collection module mainly collects and organizes the video and audio of the teaching of business administration, removes the noise part, and retains high-fidelity video and audio information; The feature extraction module is mainly divided into audio feature extraction and video feature extraction, respectively, proposes the corresponding audio feature vector and video feature vector, and then performs subsequent processing on these feature vectors; In the multimodal fusion process, the feature extraction within the modality and the feature fusion between the modalities are mainly performed, and the attention mechanism is used to complete this task.

### 3.1. Overall Network Structure

The network structure of the influence model of public mental health based on artificial intelligence technology on the teaching effect of business administration major proposed in this paper is shown in Figure 1. First of all, in order to study the effect of public mental health on the teaching of business administration majors, we need to collect video and audio data. We collected and organized the video and audio of business administration major teaching into matching data sets, namely, video content and corresponding to the audio content. Then, we use the audio feature extraction network model and the video feature extraction network model to extract features for the collected video and audio pairs, and the extracted features are expressed in the form of vectors, and then enter the next stage. Subsequently, the evaluation of school effects is carried out through public mental health based on artificial intelligence technology. In this evaluation process, the input video and audio features need to be aligned and integrated. At this stage, more attention is paid to the feature learning ability and fusion ability of the model. Finally, the teaching effect of business administration major is evaluated through the fully connected layer, and then mapped to the corresponding classification and level. In this paper, we can manually set the effect classification of learning according to actual needs. The more categories, the more accurate the classification. From these classifications, the effect of professional teaching can be evaluated.

### 3.2. Feature Extractor

In the feature extraction module, the feature extraction model of a single modality is mainly used to obtain effective information. In this paper, we need to perform feature extraction on video and audio to capture the effective information of input features. It mainly captures the in-mold feature information with the help of a single-modal GRU unit, and then process it in subsequent stages. The VGG network structure model used in this paper extracts information of different features and dimensions from left to right. This structure is similar to the spatial convolution network structure, that is, the features of the previous period can affect the characteristics of the subsequent time nodes. The method in this paper mainly considers the continuity of time and space.

In order to obtain long-term dependent relationships and contextual information of words in the input audio, we adopt Bi-GRU as the core module of the audio feature extractor. We adopt the Word2Vec pretrained model to initialize the audio feature extraction model. The formula for calculating Bi-GRU is as follows:

(1) $$\begin{array}{c} T=\left\{T_{1},T_{2},\cdots ,T_{n}\right\}, \end{array}$$

(2) $$\begin{array}{c} \overset{⟶}{h_{i}}=\overset{⟶}{\text{GRU}}\left(T_{i}\right);i\in \left[1,n\right], \end{array}$$

(3) $$\begin{array}{c} \overset{⟵}{h_{i}}=\overset{⟵}{\text{GRU}}\left(T_{i}\right);i\in \left[1,n\right], \end{array}$$

(4) $$\begin{array}{c} h_{i}=\left[\overset{⟶}{h_{i}},\overset{⟵}{h_{i}}\right];h_{i}\in R^{2k}. \end{array}$$

Equation (1) represents a text representation with *n* audio segments. For the ith time step, $\overset{⟶}{h_{i}}$ denote the hidden representation obtained by the forward GRU, $\overset{⟵}{h_{i}}$ denote the hidden representation obtained by the backward GRU, and *h*_*i*_ denote the concatenation of these two types of hidden representations. The audio feature matrix is obtained by stacking the hidden representations of *n* time steps in order.

Considering the long time and slow processing speed of video data in this paper, we first divide the video data into images of each frame, and then send them to the network for processing. We organize the collected video data, then divide the data with good video quality, select key frames from them, and then perform feature extraction on these inputs.

The image sign extraction mainly relies on the multibranch CNN-RNN module, and its network model structure is shown in Figure 2. It includes 5 CNN branch structures. The block module of each branch structure corresponds to VGG19. The feature vector extracted from each branch is passed through the convolution layer, pooling layer, and fully connected layer in turn, and finally the corresponding feature vector representation is obtained., representing the feature information from local to global. Considering that there is a strong correlation between image features at different levels and time series, for example, mid-level features are composed of bottom-level features, and high-level features are composed of mid-level features, which is a sequence relationship. In addition, there is also a correlation between the input image sequences, that is, the image of the previous frame can have an impact on the image of the subsequent frame. In this paper we employ Bi-GRU units to model the sequence dependencies of these features.

(5) $$\begin{array}{c} \overset{⟶}{l_{t}}=\overset{⟶}{\text{GRU}}\left(v_{t}\right);t\in \left[1,5\right],\\ \overset{⟵}{l_{t}}=\overset{⟵}{\text{GRU}}\left(v_{t}\right);t\in \left[1,5\right],\\ V_{m}\in R^{5\times 2k},V_{f}\in R^{2k},\\ V_{f}=\left[\overset{⟶}{l_{5}},\overset{⟵}{l_{1}}\right]. \end{array}$$

### 3.3. Multimodal Fusion

To obtain the interaction relationship between audio and image, we first use attention mechanism to obtain the correlation between different modalities, and then continuously update the text and picture feature matrix according to the learned correlation weight in Figure 3. The calculation formula of the intermodal attention mechanism is as follows:

(6) $$\begin{array}{c} \text{Attention}\left(Q,K,V\right)=\text{soft}\max\left(\frac{{QK}^{T}}{\sqrt{d}}\right)V,\\ T_{\text{update}}=\text{Attention}\left(T_{m}W_{q1},T_{m}W_{k1},T_{m}W_{v1}\right),\\ V_{\text{update}}=\text{Attention}\left(V_{m}W_{q2},V_{m}W_{k2},V_{m}W_{v2}\right). \end{array}$$

Among them, Attention() represents the operation function of the attention module; *Q*, *K*, and *V* represent the query matrix, key matrix, and value data, respectively, which is difficult; *d* is used as a scale factor, mainly to prevent the molecular dot product from being too large, and its value is input in the eigenvalues of the dimension.

The intramodal relationship is a supplement to the interaction between different modalities. In this paper, the intramodal attention mechanism module is used to model multiple single modalities, mainly to fully represent the feature information of a single modality. The calculation process is as follows:

(7) $$\begin{array}{c} T_{m2}=\text{Attention}\left(V_{m1}W_{q11},V_{m1}W_{k11},V_{m1}W_{v11}\right),\\ V_{m2}=\text{Attention}\left(V_{m1}W_{q21},V_{m1}W_{k21},V_{m1}W_{v21}\right). \end{array}$$

After performing intramodal feature representation and intermodal feature representation on multimodal data, the next step is to align and fuse multimodal data. We average pool the feature vectors obtained above, and then combine these vectors corresponds to the data label. The audio and video representations are stitched together to obtain a joint representation of the audio and video. Then, the nonlinear transformation is realized through the fully connected layer, and finally the joint representation of the multimodality is obtained, and the classification of the learning effect is carried out.

Data from different modalities, such as video and audio data, can be aligned through the attention mechanism between modalities. The attention mechanism inside the modality considers the connection between the features of the same modality data in different time and space. The aspects considered in the attention mechanism model of this paper are more comprehensive.

### 3.4. Evaluation of Teaching Effect

There is a problem of loss of video and audio information in the teaching evaluation process of business administration majors. The intramodule attention mechanism and the intermodule attention mechanism are established, and then the multimodal attention mechanism is fused. The purpose of this is to strengthen the role of the original information, while realizing the alignment of multimodal data. At the end of the model, a fully connected layer of softmax is used to map the learned high-level representations to the multiclass target space to obtain the corresponding probability distribution. We employed a cross-entropy loss function to detect the difference between the predicted probability distribution and the true labels. At the end of the network model, this paper uses the fully connected layer of softmax to map the dimensions of the final data features of the network model map. At the end of the model, it is necessary to continuously reduce the predicted probability distribution and the true probability distribution through the loss function.

## 4. Experimental Comparison and Points

### 4.1. Dataset

The teaching data set of business administration major comes from the teaching videos and audios of colleges and universities. On the basis of data collection, we organize the data sets corresponding to the videos and audios, and then classify these data sets, that is, to classify and analyze the effects of different schools. Annotation labels used to evaluate the predictive performance of the model. This paper firstly screens the data, deletes some video clips with severe noise and unclear video content in Beijing, and then trims the remaining videos to facilitate postprocessing. Then divide the dataset into a 7 : 1 : 2 ratio of training, validation, and test sets, and make sure they do not contain any of the same events.

The data collected by the method in this paper are all data from a fixed period of time. The invalid data is cleaned, and the real and valid data are completely retained. Although a lot of manpower and material resources are spent in this process, the integrity of the data is set and authenticity can be guaranteed, and human interference is reduced as much as possible.

### 4.2. Experimental Environment

The hardware environment in this article is Intel i7-8700k, 32G memory, RTX 3090 GPU, Python 3.8.8, and PyTorch 1.10. In the training of the entire network model, the batch size is set to 100, the epoch is set to 800000, the learning rate is 0.001, and the optimizer uses Adam.

### 4.3. Comparison of Experimental Results

Figure 4 represents the acquisition of video and audio data in this paper. The horizontal axis in the figure represents the number of times we collect data, and the vertical axis represents the proportion of various types of data collected. In the figure, *A*, *B*, *C*, and *D* represent four cases, such as video data, audio data, video and audio pair, and mismatched data, respectively. We can find that the video and audio pairs in the collected data are mostly used for model training and testing, and other data are deleted through data cleaning because they cannot be matched.

Figure 5 shows the proportion of dataset types in the collected data. From the figure, we can see that we divided the collated data set into five major types, namely, *A*, *B*, *C*, *D*, and *E* corresponding to the learning effect of business administration teaching: *A* means the best, and *E* grams are the worst. From the figure, we can find that most of the time, the learning effect is relatively general, and the excellent and poor are both occupying a relatively small proportion. From Figure 5, we can see that these learning effects from A to E indicate that the learning effect continues to decline: A indicates the best, E indicates the worst, and others indicate that the learning effect is moderate. We mainly classify according to the evaluation of the teachers in the class, the degree of students' participation in the classroom, and the scores through the relevant assessments. These data are relatively complete and valid data after filtering.

Figure 6 shows the training images of the proposed multimodal network model. From the figure, we can see that the *X* and *Y* axes represent the input video data and the corresponding audio data, and their positive and negative values represent increasing or decreasing the corresponding ratio. The Z-axis in the figure represents the prediction effect of the network model, and the larger the value, the higher the prediction accuracy.

Figure 7 shows the distribution map of the teaching effect of business administration majors. In the figure, *x* and *y* represent the input audio features and video features in the network, respectively, and the *z*-axis represents the distribution of the network model. From the figure we can see that the red triangles represent the number of positive samples in the network model, and the green circles represent the number of negative samples of the network model. On the whole, the positive and negative sample data of the network model are relatively balanced.

Figure 8 shows the confusion matrix of the predicted effect of the network model. The color from dark to light indicates that the prediction accuracy of learning gradually decreases. Only the case of darker color indicates that the prediction effect of the multimodal network model proposed in this paper is better. The categories 0, 1, 2, 3, 4, and 5 in the figure represent the successive declines in the effect levels of the teaching of business administration. It is also possible to expand the number of classifications of the network model according to the fine classification of other subsequent tasks, which can further subdivide this effect.

Figure 9 mainly compares the method in this paper with other evaluation methods. The horizontal axis represents the number of training times, and the vertical axis represents the prediction effect. The larger the value, the better. The other methods, Method 1, represent the multimodal network model proposed in this paper, and Methods 2 and 3 represent the use of the BERT network model and HRNet network model, respectively. This paper uses a multimodal method to extract the features of the data and realizes the multimodal data. Alignment and fusion improve the actual prediction effect of the network model.

Figure 10 shows the comparison between the method using the multimodal fusion proposed in this paper and not using the method in this paper. From the figure, we can see that the method in this paper is not used to evaluate the teaching effect of business administration, but the improvement of the effect is small, and due to the influence of human factors, it is prone to overfitting. The prediction effect of the multimodal network model proposed in this paper is relatively stable, and the prediction effect can be continuously improved with the increase of training times.

## 5. Summary

Public mental health based on artificial intelligence technology has become a key method in the field of mental health assessment. It can use artificial intelligence technology to conduct data mining and sorting technology, which can not only improve the technicality and accuracy of mental health assessment but also avoid mental health assessment. The influence of human factors in health makes mental health assessment more scientific and effective. At present, there are many methods used to evaluate the teaching effect of business administration major, and the evaluation conditions and influencing factors are many, which are easily affected by artificial factors. Evaluating the teaching effect of business administration majors from the perspective of mental health can avoid the influence of human intervention, more truly reflect the teaching status of teachers and the learning effect of students, and can effectively improve the teaching effect of business administration majors. Therefore, this paper proposes an evaluation method of public mental health based on artificial intelligence technology on the teaching effect of business administration, which avoids the influence of human operation and improves the teaching effect of business administration. At present, artificial intelligence technology is still in the stage of research and exploration, and there are many problems and deficiencies, which need to be deeply excavated and discovered according to the actual teaching of business administration. Continuous use of artificial intelligence technology plays an active role in education.

## Figures and Tables

**Figure 1:** Evaluation model of teaching effect of business administration major.

**Figure 2:** Structure diagram of feature extractor.

**Figure 3:** Multimodal fusion model.

**Figure 4:** Data set collection diagram.

**Figure 5:** Dataset type proportion diagram.

**Figure 6:** Network model training diagram.

**Figure 7:** Distribution map of teaching effect of business administration major.

**Figure 8:** Confusion matrix of network model prediction effect.

**Figure 9:** Comparison of multimethod prediction effects.

**Figure 10:** Comparison of the prediction effects of the methods in this paper.

## Data Availability

The labeled data set used to support the findings of this study is available from the corresponding author upon request.

## References

[1] Alhayani B., Mohammed H. J., Chaloob I. Z., Ahmed J. S. (2021). Effectiveness of artificial intelligence techniques against cyber security risks apply of IT industry. *Materials Today: Proceedings*.

[2] Ahmad T., Zhang D., Huang C. (2021). Artificial intelligence in sustainable energy industry: status quo, challenges and opportunities. *Journal of Cleaner Production*.

[3] Hong T., Su Q., Li X. (2021). Glucose-lowering pharmacotherapies in Chinese adults with type 2 diabetes and cardiovascular disease or chronic kidney disease. An expert consensus reported by the Chinese Diabetes Society and the Chinese Society of Endocrinology. *Diabetes/Metabolism Research and Reviews*.

[4] Ye J. M., Guo B. L., Liu Q. (2021). Clinical practice guidelines for sentinel lymph node biopsy in patients with early-stage breast cancer: Chinese Society of Breast Surgery (CSBrS) practice guidelines 2021. *Chinese Medical Journal*.

[5] Burhan Ismael N., Jabbar Othman B., Gardi B. (2021). The role of training and development on organizational effectiveness. *International Journal of Engineering, Business and Management*.

[6] Bharadwaj S., Khan N. A., Yameen M. (2021). Unbundling employer branding, job satisfaction, organizational identification and employee retention: a sequential mediation analysis. *Asia-Pacific Journal of Business Administration*.

[7] Borges A. F. S., Laurindo F. J. B., Spínola M. M., Gonçalves R. F., Mattos C. A. (2021). The strategic use of artificial intelligence in the digital era: systematic literature review and future research directions. *International Journal of Information Management*.

[8] Jianying F., Bianyu Y., Xin L., Dong T., Weisong M. (2021). Evaluation on risks of sustainable supply chain based on optimized BP neural networks in fresh grape industry. *Computers and Electronics in Agriculture*.

[9] Liu Z., Qian Q., Hu B. (2022). Government regulation to promote coordinated emission reduction among enterprises in the green supply chain based on evolutionary game analysis. *Resources, Conservation and Recycling*.

[10] Magistretti S., Ardito L., Messeni Petruzzelli A. (2021). Framing the microfoundations of design thinking as a dynamic capability for innovation: reconciling theory and practice. *Journal of Product Innovation Management*.

[11] Bashtannyk A., Akimova L. M., Kveliashvili I. M., Yevdokymov V. O., Kotviakovskyi Y. O., Akimov O. O. (2021). Legal bases and features of public administration in the budget sphere in Ukraine and foreign countries. *Ad Alta: Journal of Interdisciplinary Research*.

[12] Jaiswal A., Arun C. J. (2021). Potential of artificial intelligence for transformation of the education system in India. *International Journal of Education and Development using Information and Communication Technology*.

[13] Shorfuzzaman M., Masud M., Alhumyani H., Anand D., Singh A. (2021). Artificial neural network-based deep learning model for Covid-19 patient detection using X-ray chest images. *Engineering*.

[14] Fahim A., Addae B. A., Ofosu-Adarkwa J., Qingmei T., Bhatti U. A. (2021). Industry 4.0 and higher education: an evaluation of barriers affecting master’s in business administration enrolments using a grey incidence analysis. *IEEE Analysis Access*.

[15] Zhenghong O., Lin W., Xiaohui M. (2021). Characterization and revelation on the master program of business administration (MBA) of healthcare management in the University of Illinois at Chicago. *Chinese Journal of Medical Education*.

[16] Lai J. W., Ang C. K. E., Acharya U. R., Cheong K. H. (2021). Schizophrenia: a survey of artificial intelligence techniques applied to detection and classification. *International Journal of Environmental Research and Public Health*.

[17] Aggarwal K., Mijwil M. M., Al-Mistarehi A. H. (2022). Has the future started? The current growth of artificial intelligence, machine learning, and deep learning. *Iraqi Journal for Computer Science and Mathematics*.

[18] Zhang Z., Shi Q., He T. (2021). Artificial intelligence of toilet (AI-Toilet) for an integrated health monitoring system (IHMS) using smart triboelectric pressure sensors and image sensor. *Nano Energy*.

[19] Bressa N., Korsgaard H., Tabard A., Houben S., Vermeulen J. (2022). What's the situation with situated visualization? A survey and perspectives on situatedness. *IEEE Transactions on Visualization and Computer Graphics*.

[20] Zhong S., Zhang K., Bagheri M. (2021). Machine learning: new ideas and tools in Environmental Science and Engineering. *Environmental Science & Technology*.

[21] Kochkov D., Smith J. A., Alieva A., Wang Q., Brenner M. P., Hoyer S. (2021). Machine learning–accelerated computational fluid dynamics. *Proceedings of the National Academy of Sciences*.

[22] Perez-Vega R., Kaartemo V., Lages C. R., Borghei Razavi N., Männistö J. (2021). Reshaping the contexts of online customer engagement behavior via artificial intelligence: a conceptual framework. *Journal of Business Research*.

[23] Verma S., Sharma R., Deb S., Maitra D. (2021). Artificial intelligence in marketing: systematic review and future research direction. *International Journal of Information Management Data Insights*.

[24] Yang Z., Talha M. (2021). A coordinated and optimized mechanism of artificial intelligence for student management by college counselors based on big data. *Computational and Mathematical Methods in Medicine*.

[25] Lin S., Döngül E. S., Uygun S. V., Öztürk M. B., Huy D. T. N., Tuan P. V. (2022). Exploring the relationship between abusive management, self-efficacy and organizational performance in the context of human–machine interaction technology and artificial intelligence with the effect of ergonomics. *Sustainability*.

[26] Klos M. C., Escoredo M., Joerin A., Lemos V. N., Rauws M., Bunge E. L. (2021). Artificial intelligence–based chatbot for anxiety and depression in university students: pilot randomized controlled trial. *JMIR Formative Research*.

[27] Mengi M., Malhotra D. (2021). Artificial intelligence based techniques for the detection of socio-behavioral disorders: a systematic review. *Archives of Computational Methods in Engineering*.

[28] Lin Q., Li T., Shakeel P. M., Samuel R. D. J. (2021). Advanced artificial intelligence in heart rate and blood pressure monitoring for stress management. *Journal of Ambient Intelligence and Humanized Computing*.

